# Piperlongumine inhibits lung tumor growth via inhibition of nuclear factor kappa B signaling pathway

This article has been retracted.

**DOI:** 10.1038/srep26357

**Published:** 2016-05-20

**Authors:** Jie Zheng, Dong Ju Son, Sun Mi Gu, Ju Rang Woo, Young Wan Ham, Hee Pom Lee, Wun Jae Kim, Jae Kyung Jung, Jin Tae Hong

**Affiliations:** 1 College of Pharmacy and Medical Research Center, Chungbuk National University, Osong-eup, Heungduk-gu, Cheongju, Chungbuk 28160, Republic of Korea; 2 New Drug Development Center, KBio, Osong-eup, Heungduk-gu, Cheongju, Chungbuk 28160, Republic of Korea; 3 Department of Chemistry, Utah Valley University, 800 West University Parkway, Orem, UT 84508, USA; 4 College of Medicine, Chungbuk National University, Chungdae-ro 1, Seowon-gu, Cheongju, Chungbuk 28644, Republic of Korea

## Abstract

Piperlongumine has anti-cancer activity in numerous cancer cell lines via various signaling pathways. But there has been no study regarding the mechanisms of PL on the lung cancer yet. Thus, we evaluated the anti-cancer effects and possible mechanisms of PL on non-small cell lung cancer (NSCLC) cells *in vivo* and *in vitro*. Our findings showed that PL induced apoptotic cell death and suppressed the DNA binding activity of NF-κB in a concentration dependent manner (0–15 μM) in NSCLC cells. Docking model and pull down assay showed that PL directly binds to the DNA binding site of nuclear factor-κB (NF-κB) p50 subunit, and surface plasmon resonance (SPR) analysis showed that PL binds to p50 concentration-dependently. Moreover, co-treatment of PL with NF-κB inhibitor phenylarsine oxide (0.1 μM) or p50 siRNA (100 nM) augmented PL-induced inhibitory effect on cell growth and activation of Fas and DR4. Notably, co-treatment of PL with p50 mutant plasmid (C62S) partially abolished PL-induced cell growth inhibition and decreased the enhanced expression of Fas and DR4. In xenograft mice model, PL (2.5–5 mg/kg) suppressed tumor growth of NSCLC dose-dependently. Therefore, these results indicated that PL could inhibit lung cancer cell growth via inhibition of NF-κB signaling pathway *in vitro* and *in vivo*.

Lung cancer is the leading cause of cancer death and the second most common cancer among both men and women in the United States^1^. An estimated 224210 new cases in the United States will be diagnosed with lung cancer^1^. There are two major types of lung cancer. One is small cell lung cancer (SCLC) and the other is non-small cell lung cancer (NSCLC). About 85% to 90% lung cancers are NSCLC^2^. Current treatments such as surgery, radiotherapy and chemotherapy have been used for treating lung cancer patients^3^. But these treatments are not sufficient and progress of resistance against chemotherapy, toxicity and side-effects is still a main obstacle. Thus, it is urgent to develop novel anti-cancer agents with little side effects and toxicities.

Numerous evidences showed that constitutive activation of nuclear factor kappa B (NF-κB) is often found in human cancer cells including non-small cell lung cancer tissue and cell lines^4^. Tumor samples obtained from lung cancer patients showed high levels of NF-κB activation in both SCLC and NSCLC^4^,^5^. NF-κB plays a vital role in the suppression of apoptosis and in the induction of proliferation, inflammation and cancer development^6^. NF-κB acts as a cell survival factor via regulating the expression of an array of apoptotic (caspase-3 and Bax), anti-apoptotic (Bcl-2 and IAP family) and cell proliferation genes (cyclooxygenase-2 and cyclins)^7^. It has been reported that numbers of anti-cancer natural compounds inhibit the growth of NSCLC cells via NF-κB signaling pathway. Protocatechuic acid inhibits lung cancer cells by modulating p-focal adhesion kinase (FAK), mitogen-activated protein kinase (MAPK) and NF-κB pathways^8^. Theanine derivatives inhibit lung tumor growth by targeting epidermal growth factor receptor (EGFR)/vascular endothelial factor receptor (VEGFR)-Akt/NF-κB pathways^9^. Our previous study also demonstrated that several compounds such as bee venom, thiacremonone and (E)-2,4-bis (*p-*hydroxyphenyl)-2-butenal showed anti-cancer activity via inhibition of NF-κB in NSCLC cells^10^,^11^,^12^.

Piperlongumine (PL), a natural product isolated from the long pepper *piper longum* L.^13^, was recently identified as selectively toxic to cancer cells *in vitro* and *in vivo*^14^. PL has anti-cancer activity in colon, ovarian, prostate, breast, pancreatic, head and neck and renal cancer via multiple signaling pathways^15^,^16^,^17^,^18^,^19^,^20^,^21^. However, there has been no study regarding the mechanisms of PL on the lung cancer yet. Notably, in prostate cancer, PL inhibited cancer cell growth via inhibition of NF-κB^20^. Thus, in this study, we evaluated the anti-cancer effects and possible mechanisms of PL on NSCLC cells *in vivo* and *in vitro*.

## Results

### PL is expected to have high drug-likeness

To investigate whether PL has high drug-likeness properties to be developed as a medicine, we have performed an *in silico* ADME and toxicology studies. *In silico* ADME analysis, PL showed high human intestinal absorption (HIA) and blood-brain barrier (BBB) penetration levels (Table 1) which are major properties of promising drugs^22^. Through *in silico* toxicity analysis, we observed that PL is predicted to be markedly little toxic (Table 2). Taken together, these results suggested that PL might have low toxicity and excellent ADME profiles which are great advantages in drug development.

### Effect of PL on the growth of NSCLC cells and lung epithelial cells

To evaluate the effect of PL on the growth of lung cancer and normal cells, we analyzed cell viability using the MTT assay. PL (0–20 μM) inhibited the growth of A549 and NCI-H460 NSCLC cells, but showed no significant effect on LL-24 lung epithelial normal cells (Fig. 1a), and IC_50_ values of A549 and NCI-H460 were 14.91 μM and 13.72 μM, respectively (Fig. 1b). To determine whether the cell growth inhibition by the PL was due to the induction of apoptosis, we evaluated the changes in NSCLC cells by using DAPI staining followed by TUNEL assay, and then the double labeled cells were analyzed by fluorescence microscope. The cells were treated with concentrations of PL (0–20 μM) for 24 h. DAPI-stained TUNEL-positive cells were concentration-dependently increased (Fig. 1c) and the highest concentration of PL (20 μM) caused most of cells TUNEL-positive, and apoptosis rates were 62.59% in A549 cells and 66.36% in NCI-H460 cells (Fig. 1d). These results demonstrated that PL strongly induced apoptotic cell death in NSCLC cells.

### Effect of PL analogues on the growth of A549 NSCLC cells and on NF-κB luciferase activities

To find out the best compound which exhibits anti-cancer effect in NSCLC cells, we performed cell proliferation assay in A549 cells. We tested 36 PL analogues in the present study (structure shown in Supplementary Fig. 1a,b). Of all 37 compounds, PL showed the most significant cell growth inhibitory effect in A549 cells (Supplementary Fig. 2a). We also performed luciferase assay to assess NF-κB binding affinities in A549 cells (Supplementary Fig. 2b). Interestingly, PL also showed the best inhibitory effect on NF-κB activity in A549 cells (Table 3), suggesting that it is possible to evaluate anti- cancer effect of PL by targeting NF-κB signaling pathway. Notably, both compounds 21 and 22 showed NF-κB inhibitory effect as similar as PL, but did not show cell growth inhibitory effect as similar as PL. It may due to unknown cell death signaling that could be regulated by PL.

### Effect of PL on the expression of apoptosis regulatory proteins

To figure out the relationship between the induction of apoptosis and the expression of apoptosis regulatory proteins by PL treatment, the expression of apoptosis regulatory proteins was investigated. When treated with PL (0–15 μM) in A549 and NCI-H460 NSCLC cells, we found that the expression of various apoptotic proteins such as Bax, cleaved caspase-3, cleaved caspase-8 was increased, while the expression of anti-apoptotic protein Bcl-2 was decreased in a concentration dependent manner (Fig. 2a,b). NSCLC cells were treated with non-targeting control siRNA and Fas, DR3, DR4, DR5, DR6 siRNA (100 nM) for 24 h, and then were treated with PL (10 μM) for another 24 h. Cell viability was determined by MTT assay. Expression of Fas and DR4 was increased in a concentration dependent manner (0–15 μM) in A549 (Fig. 2c) and NCI-H460 (Fig. 2d) NSCLC cells.

### Effect of PL on the DNA binding activity of NF-κB

NF-κB plays a pivotal role in cancer cell survival. To investigate whether PL inactivates NF-κB, we performed EMSA for detecting DNA binding activity of NF-κB. We found that PL non-treated NSCLC cells showed highly constituted activation of NF-κB in both cancer cells. However, PL treatment concentration dependently inhibited DNA binding activity of NF-κB in A549 (Fig. 3a) and NCI-H460 cells (Fig. 3b). Besides, Luciferase assay was carried out to confirm the effect of PL on NF-κB activity. We found that PL reduced NF-κB luciferase activity in a concentration dependent manner in A549 (Fig. 3c) and NCI-H460 cells (Fig. 3d).

Expression levels of cytosol extracted proteins IκBα and p-IκBα and nucleus extracted proteins p50 and p65 were determined by Western blotting. We found that the expression of p-IκBα and the nuclear expression of p50 and p65 was decreased in A549 (Fig. 3e) and NCI-H460 cells (Fig. 3f).

### Combination effect of PL with p50 siRNA transfection or NF- κB inhibitor on PL-induced cell growth inhibition and expression of Fas and DR4

To investigate whether NF-κB plays a critical role in PL-induced NSCLC cell growth inhibition, we pretreated the NSCLC cells with NF-κB inhibitor PAO (0.1 μM for 1 h, and then these cells were treated with PL (10 μM) for 24 h to assess cell viability. As a result, co-treatment with PL and PAO augmented PL-induced cell growth inhibition (Fig. 4a), and magnified the enhanced expression of Fas and DR4 (Fig. 4b). To further determine the relationship between NF-κB activity and NSCLC cell growth inhibitory effect of PL, A549 and NCI-H460 cells were transfected with p50 siRNA using a transfection agent for 24 h, and then treated with PL (10 μM) for 24 h. Co-treatment with PL and p50 siRNA transfection also augmented PL-induced cell growth inhibition in A549 and NCI-H460 (Fig. 4c) and enhanced the expression of Fas and DR4 (Fig. 4d). These data suggested that NF-κB pathway may be involved in PL-induced cell growth inhibition.

### Reversed effect of p50 mutant plasmid (C62S) on PL-induced cell growth inhibition and expression of Fas and DR4

The sulphydryl group of Cys62 is an important determinant of DNA recognition by p50 subunit of NF-κB^23^. To further demonstrate the pivotal role of NF-κB on PL-induced cell growth inhibition, we performed mutant plasmid construction assay. A549 and NCI-H460 NSCLC cells were transfected with p50 mutant plasmid (C62S) for 24 h, and then were treated with PL (10 μM) for another 24 h. As a result, p50 mutant plasmid (C62S) partially abolished PL-induced cell growth inhibition (Fig. 5a), and partially prevented enhanced expression of Fas and DR4 (Fig. 5b).

### Reversed effect of Fas siRNA and DR4 siRNA transfection on PL-induced cell growth inhibition and DNA binding activity of NF-κB

To confirm the importance of DRs on PL-induced cell death, we performed MTT assay and siRNA transfection. Effect of Fas siRNA or DR4 siRNA on the expression of each DR was evaluated by Western blotting. The expression of Fas or DR4 was knocked down by each siRNA (Supplementary Fig. 3). Knock down of Fas or DR4 partially abolished PL-induced cell growth inhibition rather than DR3, DR5 and DR6 (Fig. 5c). Notably, Fas siRNA and DR4 siRNA transfection also partially abolished PL-induced inhibition of DNA binding activity of NF-κB in A549 and NCI-H460 NSCLC cells (Fig. 5d).

### Structure of PL and molecular binding between PL and p50

The molecular binding between PL (Fig. 6a) - p50 protein was assessed using pull-down assay. The interaction of PL-Sepharose 4B beads with p50 was then detected by immunoblotting with p50 antibody. The results indicated that PL bound with cell lysates containing p50 from SW480 cells and p50 recombinant protein (Fig. 6b). Surface Plasmon resonance (SPR) assay also showed that PL bound to p50 recombinant protein in a concentration dependent manner (31.25–500 μM) (Fig. 6c). To identify the binding site of PL to p50, we performed computational docking experiments with PL and p50. PL directly bound in a pocket of NF-κB p50 subunit (created by Phe353, Arg356, Gly361, Ser363, His364, Gly365, Val412, Gly413, Lys414, Asn436, Gly438, Lle439 and Leu440) next to the DNA binding site (Fig. 6d,e).

### Effect of PL on lung cancer tumor growth

To elucidate the anti-tumor effect of PL *in vivo*, the tumor growth on lung cancer cell xenograft bearing nude mice following PL treatments was investigated. In A549 xenograft studies, PL was administrated intraperitoneally twice per week for 3 weeks to mice which have tumors ranging from 100–150 mm^3^. Tumor volume was measured weekly, and all mice were sacrificed at the end of experiment when tumors were dissected and weighted. The inhibitory effect of PL on the growth of lung tumor was significant in xenograft model mice (Fig. 7a). Tumor volume and weight were dose-dependently decreased (Fig. 7b,c). The immunohistochemistry analysis of tumor section by hematoxylin and eosin staining revealed that PL dose-dependently inhibited tumor growth, and the expression level of active caspase-3 was increased while the expression level of p50 was decreased in nude mice xenograft tissues. To determine whether the cell growth inhibition by the PL was due to the induction of apoptosis *in vivo*, we evaluated the changes in xenograft tumor tissues by using DAPI staining followed by TUNEL assay, and then the double labeled tissues were analyzed by fluorescence microscope. As a result, PL induced apoptosis in a dose dependent manner (2.5–5 mg/kg) (Fig. 7d).

### Effect of PL on the expression of apoptosis regulatory proteins and on the DNA binding activity of NF-κB in lung tumor tissues

To evaluate the effect of PL on the expression of apoptosis regulatory proteins, we performed Western blotting analysis. The results showed that the expression of Fas and DR4 was increased (Fig. 8a), and the expression of cleaved caspase-3, cleaved caspase-8 and Bax was increased while the expression of Bcl-2 was decreased in a dose dependent manner (Fig. 8b). We also found the DNA binding activity of NF-κB was decreased in a dose dependent manner (2.5–5 mg/kg) in lung tumor tissues (Fig. 8c) and the nuclear expression of p50 and p65 was decreased (Fig. 8d).

## Discussion

Recent studies on the signaling mechanisms of DRs have revealed that members of caspase families are key regulators of cell death. Expression of DRs lead to activation of caspase signaling pathway to induce apoptotic cell death^24^. In our present study, we found that PL induced apoptotic cell death through activation of Fas and DR4. It was also found that these effects were correlated with the enhanced expression of apoptotic proteins such as Bax, cleaved caspase-3 and cleaved caspase-8 in a concentration dependent manner (0–15 μM). However, the expression of anti-apoptotic protein Bcl-2 was decreased. It was reported that numerous natural compounds showed anti-cancer effect via activation of DRs recently. In our previous study, we presented that BV suppressed cancer cell growth via activation of DR3 in NSCLC cells^10^, Myriocin induced apoptotic cell death through activation of DR4 in NSCLC cells^25^, (E)-2,4-bis (p-hydroxyphenyl)-2-butenal showed anti-cancer effect via activation of DR5 in NSCLC cells^12^. Our findings also showed that knock down of Fas or DR4 with siRNA partially abolished the inhibitory effect of PL on the NSCLC cell growth. Besides, co-treatment with PL and p50 siRNA transfection or phenylarsine oxide (PAO) magnified the PL-induced enhanced expression of Fas and DR4. These data demonstrated that PL-induced apoptotic cell death was correlated with enhanced expression of Fas and DR4.

Constitutive activation of NF-κB is often found in human cancer cells including non-small cell lung cancer tissue and cell lines^4^. Tumor samples obtained from lung cancer patients showed high levels of NF-κB activation in both SCLC and NSCLC^4^,^5^. It was demonstrated that NF-κB acts as a cell survival factor via regulation with apoptotic, anti-apoptotic and cell proliferation genes^7^. PL treatment suppressed the DNA binding activity of NF-κB, phosphorylation of IκBα and nuclear translocation of p50 and p65 in a concentration dependent manner (0–15 μM). We performed pull-down assay to confirm that PL binds to NF-κB p50 subunit. Besides, SPR analysis also showed that PL binds to NF-κB p50 in a concentration dependent manner (31.25–500 μM). Docking experiment showed that PL directly binds in a pocket of NF-κB p50 subunit (created by Phe353, Arg356, Gly361, Ser363, His 364, Gly365, Val412, Gly413, Lys414, Asn436, Gly438, Lle439 and Leu440) next to the DNA binding site which may interrupt with DNA binding event. Similar mechanism was found in the inhibitory effect on cancer cell growth of thiacremonone and tectochrysin that bound to the DNA binding site of p50 to inhibit the DNA binding activity of NF-κB in NSCLC cells^26^,^27^. Besides, (E)-2,4-Bis (*p*-hydroxyphenyl)-2-butenal inhibits NF-κB activity via directly binding to IKKβ^28^, (E)-4-(3-(3,5-dimethoxyphenyl)allyl)-2-methoxyphenol inhibits NF-κB activity via directly binding to DNA binding site of p50^29^. Melittin, the major component of bee venom directly bound to the nuclear localization sequence (NLS) which was near to the C-terminus of p50 to block NF-κB activation^30^. With agreement of this notion, our findings also showed that p50 mutant plasmid (C62S) where the cysteine residue at 62 of p50 was replaced by serine partially abolished PL-induced cell growth inhibition. Thus, it suggested that PL showed anti-cancer effect via modulation of cysteine residues of NF-κB p50 subunit.

The studies on the signaling mechanisms of DRs have also revealed that NF-κB is key regulator of apoptotic cells death. NF-κB directly regulates Fas transcription to modulate Fas-mediated apoptosis and tumor suppression^31^. Numerous studies have demonstrated that the anti-cancer compound targeting NF-κB leads to DR-induced apoptotic cell death. Our previous study also showed that bee venom inhibited NSCLC cell growth via activation of DR3 and inhibition of NF-κB^10^. (E)-2,4-bis (p-hydroxyphenyl)-2-butenal showed anti-proliferative effect via MAPK-mediated suppression of NF-κB and up-regulation of DR5^12^. Moreover, co-treatment with PL and p50 siRNA transfection or NF-κB inhibitor PAO augmented the cell growth inhibition in NSCLC cells. PL could suppress NF-κB activity while p50 siRNA itself could suppress the expression of p50, and PAO may suppress the phosphorylation of IκBα. Thus, co-treatment with PL and p50 siRNA transfection or PAO may augment PL-induced inhibition of NF-κB activity to induce more apoptotic cell death. Notably, p50 mutant plasmid (C62S) transfection partially abolished PL-induced cell growth inhibition, and decreased PL-induced enhanced expression of Fas and DR4. These data indicated that PL inhibited the NSCLC cell growth via preventing nuclear translocation of NF-κB p50 subunit to suppress the DNA binding activity of NF-κB. In addition, it was demonstrated that NF-κB directly up-regulates anti-apoptotic proteins such as C-FLIP which is a specific inhibitor of caspase-8 to block activation of caspase-8 that could be induced by DR signaling^32^. Moreover, inhibition of NF-κB by several chemotherapeutics exposures human cancer cells to induction of apoptosis via up-regulation of DRs^33^. Thus, it is possible that PL induces apoptotic cell death via inhibition of NF-κB, resulting in induction of Fas and DR4.

To further demonstrate the anti-cancer effects, we performed animal experiments with xenograft nude mice model. The present data showed that PL suppressed lung tumor growth, tumor volume and tumor weight in a dose dependent manner (2.5–5 mg/kg). Besides, Western blotting data showed that the expression of apoptotic proteins such as Bax, cleaved caspase-3, cleaved caspase-8, Fas and DR4 was increased while the expression of anti-apoptotic protein Bcl-2 was decreased in a dose dependent manner (2.5–5 mg/kg). The immunohistochemistry analysis also showed that the expression level of active caspase-3, Fas and DR4 was increased while the expression level of PCNA and NF-κB p50 subunit was decreased in a dose dependent manner (2.5–5 mg/kg). Moreover, the DNA binding activity of NF-κB was also decreased in a dose dependent manner (2.5–5 mg/kg). In addition, we also found that PL induced apoptosis in xenograft tumor tissues in a dose dependent manner (2.5–5 mg/kg). These data indicated that PL could directly block NF-κB activation to induce Fas and DR4 mediated apoptotic cell death showing anti-cancer effect in NSCLC cells *in vivo* and *in vitro*.

In addition, our predicted ADME and toxicities of PL showed that PL has excellent drug-likeness, permeability and solubility with low toxicities. Notably, prediction of blood-brain barrier (BBB) penetration and human intestinal absorption (HIA) is one of major goals for selection of candidates, drug design and drug development^22^. In our analysis results, PL showed high HIA and BBB penetration levels. Moreover, we have performed cell proliferation assay and NF-κB luciferase assay with PL and 36 PL analogues. As a result, we found that PL showed the most significant cell growth inhibitory effect and the best NF-κB binding affinity. In conclusion, PL could inhibit lung tumor growth via activation of Fas and DR4, and inhibition of NF-κB signaling pathway *in vivo* and *in vitro*. Because PL is selectively toxic to cancer cells with high drug-likeness and permeability, it may be a promising anti-cancer agent with little side effect for treatment of lung cancer.

## Materials and Methods

### Materials

Caspase-3, caspase-8 antibodies were purchased from Cell Signaling Technology Inc. (Beverly, MA). Bcl-2, Bax, p50, p65, Histone-H1 and β-actin antibodies were purchased from Santa Cruz Biotechnology, Inc. (Santa Cruz, CA). The cell culture materials were obtained from GIBGO^®^ of Introgen™ (Seoul, Korea), and other chemical reagents were from Sigma Chemical Co.

### Cell culture

A549 and NCI-H460 NSCLC cells and LL-24 lung epithelial cells were obtained from American Type Culture Collection (ATCC, Manassas, VA, USA). A549 and NCI-H460 cells were cultured in RPMI 1640 medium supplemented with 10% heat inactivated fetal bovine serum (FBS), 100 units/ml penicillin and 100 μg/ml streptomycin (Invitrogen). LL-24 cells were cultured in DMEM medium supplemented with 10% heat inactivated FBS, 100 units/ml penicillin and 100 μg/ml streptomycin (Invitrogen). Cell cultures were then maintained in an incubator within a humidified atmosphere of 5% CO_2_ at 37 °C.

### Cell viability assay

A549 and NCI-H460 NSCLC cells were plated in 96-well plates, subsequently treated with PL (0–20 μM) for 24 h. After treatment, cell viability was measured by MTT [3-(4, 5-Dimethylthiazol-2-yl)-2, 5-Diphenyltetrazolium Bromide] assay (Sigma Aldrich, St. Louis, MO) according to the manufacturer’s instructions. Briefly, MTT (5 mg/mL) was added and plates were incubated at 37 °C for 4 h before dimethyl sulfoxide (100 μL) was added to each well. Finally, the absorbance of each well was read at a wavelength of 540 nm using a plate reader.

### Detection of Apoptosis

A549 and NCI-H460 NSCLC cells were cultured on 8-chamber slides and washed twice with phosphate buffered saline (PBS) and fixed by incubation in 4% paraformaldehyde in PBS for 1 h at room temperature. TdT-mediated dUTP nick and labeling (TUNEL) assays were performed by using the DeadEnd™ Fluorometric TUNEL System (Promega, Madison, USA) according to manufacturer’s instructions. Total number of cells in a given area was determined by using DAPI staining. The apoptotic index was determined as the number of TUNEL-positive stained cells divided by the total cell number counted x100%.

### Western blotting

A549 and NCI-H460 NSCLC cells treated with PL (0–20 μM) for 24 h were homogenized with a protein extraction solution (PRO-PREPTM, Intron Biotechnology), and lysed by 60 min incubation on ice. The cell lysate was centrifuged at 13,000 rpm for 15 min at 4 °C. Equal amount of proteins (40 μg) were separated on a SDS/12%-polyacrylamide gel, and then transferred to a polyvinylidene fluoride (PVDF) membrane (GE Water and Process technologies). Blots were blocked for 1 h at room temperature with 5% (w/v) non-fat dried milk in Tris-Buffered Saline Tween-20 [TBST: 10 mM Tris (pH 8.0) and 150 mM NaCl solution containing 0.05% Tween-20]. After a short washing in TBST, the membranes were immunoblotted with the following primary antibodies: caspase-3, caspase-8 (1:1000 dilutions; Cell Signaling, Beverly, MA) and Bcl-2, Bax and β-actin (1:1000 dilutions; Santa Cruz Biotechnology, Santa Cruz, CA). The blots were performed using specific antibodies followed by second antibodies and visualization by chemiluminescence (ECL) detection system.

### Electrophoretic mobility shift assay

The DNA binding activity of NF-κB was determined using an electrophoretic mobility shift assay (EMSA) performed as according to the manufacturer’s recommendations (Promega, Madison, USA). The relative densities of the DNA–protein binding bands were scanned by densitometry using MyImage (SLB), and quantified by Labworks 4.0 software (UVP, Inc., Upland, CA).

### Transfection of siRNA

A549 and NCI-H460 NSCLC cells were plated in 6-well plates (2 × 10^5^ cells/well) and were transiently transfected with siRNA, using a mixture of siRNA and Lipofectamine 3000 reagent in OPTI-MEM, according to the manufacturer’s specification (Invitrogen, Carlsbad, CA, USA). The transfected cells were treated with PL (10 μM) for 24 h and then used for detecting cell viability and protein expression.

### Luciferase assay

A549 and NCI-H460 cells were plated in 12-well plates (1 × 10^5^ cells/well) and transiently transfected with pNF-κB-Luc plasmid (5× NF-κB; Stratagene, La Jolla, CA, USA) using a mixture of plasmid and Lipofectamine 3000 in OPTI-MEM according to manufacturer’s specification (Invitrogen, Carlsbad, CA, USA) for 24 h. The transfected cells were treated with PL for another 24 h. Luciferase activity was measured by using the luciferase assay kit (Promega, Madison, USA), and the results were read on a luminometer as described by the manufacturer’s specifications (WinGlow, Bad Wildbad, Germany).

### Antitumor activity study in *in vivo* xenograft animal model

Seven-week-old male BALB/C nude mice were purchased from Orient-Bio (Gyunggi-do, Korea). The mice were maintained in accordance with the Korea Food and Drug Administration guidelines as well as the regulations for the care and use of laboratory animals of the animal ethics committee of Chungbuk National University (CBNU-278-11-01). A549 NSCLC cells were injected subcutaneous (1 × 10^7^ tumor cells/0.1 ml PBS/animals) with a 27-gauge needle into the right lower flanks in carrier mice. After 10–14 days, when the tumors had reached an average volume of 100–150 mm^3^, the tumor-bearing nude mice were intraperitoneally (i.p.) injected with PL (2.5 mg/kg and 5 mg/kg dissolved in 0.01% DMSO) twice per week for 3 weeks. The group treated with 0.01% DMSO was designed as the control. The weight and tumor volume of the animals were monitored twice per week. The tumor volumes were measured with vernier calipers and calculated by the following formula: (A × B^2^)/2, where A is the larger and B is the smaller of the two dimensions. At the end of the experiment, the animals were sacrificed with cervical dislocation. The tumors were separated from the surrounding muscles and dermis, excised and weighed.

### Immunohistochemistry

The animal tissues were fixed in 4% paraformaldehyde and cut into 5 μm sections using a freezing microtome (Thermo Scientific, Germany). The sections were stained with hematoxylin and eosin (H&E) for pathological examination. For immunohistological staining, tumor sections were incubated with primary antibody against PCNA, Fas, DR4, p50, active caspase-3 (1:500, Abcam, Cambridge, UK). After rinse in phosphate buffered saline (PBS), the sections were subject to incubation in biotinylated secondary antibody. The tissue was incubated for 1 h in an avidin-peroxidase complex (ABC, Vector Laboratories, Inc., Burlingame, CA). After washing in PBS, the immunocomplex was visualized using 3, 3-diaminobenzidine solution (2 mg/10 ml) containing 0.08% hydrogen peroxide in PBS. Sections were dehydrated in a series of graded alcohols, cleared in xylene and coverslipped using Permount (Fisher Scientific, Suwanee, GA).

### Pull-down assay

PL was conjugated with epoxy-activated Sepharose4B. PL (1 mg) was dissolved in 1 ml of coupling buffer (0.1 M NaHCO_3_, pH 8.3 containing 0.5 M NaCl). The epoxy-activated Sepharose 4B was swelled and washed in distilled water on a sintered glass filter, then washed with the coupling buffer. Epoxy-activated Sepharose4B beads were added to the PL-containing coupling buffer and rotated at 4 °C for overnight. After washing, unoccupied binding sites were blocked with 0.1 M Tris-HCl buffer (pH 8.0) 2 h at room temperature. The PL-conjugated Sepharos4B was washed with three cycles of alternating pH wash buffers (buffer 1: 0.1 M acetate and 0.5 M NaCl, pH 4.0; buffer 2: 0.1 M Tris-HCl and 0.5 M NaCl, pH 8.0). The control unconjugated epoxy-activated Sepharose4B beads were prepared as described above in the absence of PL. The cell lysate was mixed with PL-conjugated Sepharose4B or Sepharose4B at 4 °C for overnight. The beads were then washed on time with TBST. The bound proteins were eluted with SDS loading buffer. The proteins were then resolved by SDS-PAGE followed by immunoblotting with antibodies against p50 (1:1000 dilutions, Santa Cruz Biotechnology, Santa Cruz, CA).

### Docking experiment

Docking studies between NF-κB p50 subunit and PL was performed using Autodock VINA^34^. Only one monomer of the homo-dimeric p50 crystal structure was used in the docking experiments and conditioned using AutodockTools by adding all polar hydrogen atoms. Three dimensional structures of p50-DNA complexes were retrieved from the Protein Data Bank (PDB codes: 1VKX). Starting from the co-crystallized complexes, the p50 monomer chain (p50 from 1VKX), PL for docking were prepared using Maestro graphical interface. The grid box was centered on the p50 monomer and the size of the grid box was adjusted to include the whole monomer. Docking experiments were performed at various exhaustiveness values of the defaults: 16, 24, 32, 40 and 60. Molecular graphics for the best binding model was generated using Discovery Studio Visualizer 2.0.

### Surface Plasmon resonance (SPR) analysis

Biacore T200 and CM5 sensor chip were both supplied by GE healthcare (Uppsala, Sweden). Recombinant protein p50 of NF-κB subunit were purchased from Cayman Chemical (Ann Arbor, MI, USA). GST-fused p50 was immobilized in CM5 chip by amine coupling method. Immobilized level were reached in 12000 RU corresponded to R_max_ = 50 RU at 10 mM Na acetate pH 4.0. Binding sensorgram were detected with PL (31.25, 62.5, 125, 250 and 500 μM in 1X PBS, 5% DMSO) at 25 °C. To eliminate DMSO effect was achieved solvent correction. Sensorgram was evaluated with Biacore T 200 Evaluation software ver 1.0. The response curves with various analyze concentration were fitted with 1:1 (langmurie) binding model.

### Prediction of drug-likeness

We carried out an *in silico* toxicology and ADME (absorption, distribution, metabolism, and extraction) evaluation by using computational ADME QSAR models, preADMET (http://preadmet.bmdrc.org) and StarDrop (http://www.optibrium.com/stardrop/stardrop-features.php), to predicted the major toxicities and ADME of PL.

### Statistical analysis

All statistical analysis was performed with GraphPad Prism 5 software (Version 5.0, GraphPad Software, Inc., San Diego, CA, USA). Group differences were analyzed using two-way analysis of variance (ANOVA) followed by Tuckey’s test or one-way ANOVA followed by Dunnett’s test. All values are presented as mean ± S.D. Significance was set at *p* < 0.05 for all tests.

## Additional Information

**How to cite this article**: Zheng, J. *et al*. Piperlongumine inhibits lung tumor growth via inhibition of nuclear factor kappa B signaling pathway. *Sci. Rep.* **6**, 26357; doi: 10.1038/srep26357 (2016).

## Supplementary Material

Supplementary Information

## Figures and Tables

**Figure 1:** Effect of PL on the growth of NSCLC cells and lung epithelial cells, and effect of PL on apoptotic cell death in NSCLC cells. Concentration-dependent inhibitory effect of PL on cancer cell growth was found in A549 and NCI-H460 NSCLC cells but not in LL-24 cells. (**a**) Morphological changes of A549 and NCI-H460 NSCLC cells and LL-24 lung epithelial cells were observed under phase contrast microscope. (**b**) Relative cell survival rate was determined by MTT assay. Data was expressed as the mean ± S.D. of three experiments. *p < 0.05 indicates significant difference from control group. (**c**) Apoptotic cell death of A549 and NCI-H460. NSCLC cells were treated with PL (0–20 μM) for 24 h, and then labeled with DAPI and TUNEL solution. Total number of cells in a given area was determined by using DAPI nuclear staining (fluorescent microscope). A green color in the fixed cells marks TUNEL-labeled cells. (**d**) Apoptotic index was determined as the DAPI-stained TUNEL-positive cell number/total DAPI-stained cell number x 100%. Data was expressed as the mean ± S.D. of three experiments. *p < 0.05 indicates significant difference from control group.

**Figure 2:** Effect of PL on the expression of apoptosis regulatory proteins in NSCLC cells. (**a**,**b**) Expression of apoptosis regulatory proteins was determined by Western blotting with antibodies against cleaved capase-3, cleaved caspase-8, Bax, Bcl-2 and β-actin (internal control). Each band is representative for three experiments. (**c,d**) Expression of Fas and DR4 was determined by Western blotting. For the cropped images, samples were run in the same gels under same experimental conditions and processed in parallel. Each band is representative for three experiments. Full-length gels are presented in Supplementary Fig. 4.

**Figure 3:** Effect of PL on the DNA binding activity of NF-κB. (**a,b**) NSCLC cells were treated with PL (0–15 μM) for 2 h, and then were lysed with A buffer and C buffer. Nuclear extracts were incubated in binding reactions of ^3^^2^p-end-labeled oligo nucleotide containing the NF-κB sequence. The present EMSA results are representative for three experiments. (**c,d**) NSCLC cells were tranfected with pNF-κB-Luc plasmid for 24 h. The transfected cells were treated with PL (0–15 μM) for another 24 h. Luciferase activity was measured by using the luciferase assay kit. The present results are representative for three experiments. (**c**,**d**) Cytosol proteins were used to determine the expression of IκBα, p-IκBα and β-actin (internal control) in NSCLC cells. Nuclear proteins were used to determine the expression of p50, p65 and Histone H1 (internal control) in NSCLC cells. For the cropped images, samples were run in the same gels under same experimental conditions and processed in parallel. Each band is representative for three experiments. Full-length gels are presented in Supplementary Fig. 5.

**Figure 4:** Effect of p50 siRNA transfection or NF-κB inhibitor on PL-induced cell growth inhibition and expression of Fas and DR4 in NSCLC cells. (**a**) Cells were pretreated with NF-κB inhibitor, PAO (0.1 μM) for 1 h and then were treated with PL for 24 h. Cell viability was determined by MTT assay. Data was expressed as the mean ± S.D. of three experiments. *p < 0.05 indicates significantly different from control cells. ^#^*p* < 0.05 indicates significantly different from PL-treated cells. (**b**) Effect of NF-κB inhibitor (PAO) on the expression of death receptors. Cells were pretreated with PAO (0.1 μM) for 1 h and then were treated with PL for 24 h, and whole cell extracts were analyzed by Western blotting using Fas, DR4 and β-actin (internal control). Each band is representative for three experiments. (**c**) NSCLC cells were treated with non-targeting control siRNA and p50 siRNA (100 nM) for 24 h, and then were treated with PL (10 μM) for another 24 h. Cell viability was determined by MTT assay. Data was expressed as the mean ± S.D. of three experiments. *p < 0.05 indicates statistically significant differences from control cells. ^#^*p* < 0.05 indicates significantly different from PL treated cells. (**d**) Effect of p50 knockdown on the expression of death receptors was determined by using Western blotting with antibodies against Fas, DR4 and β-actin (internal control). For the cropped images, samples were run in the same gels under same experimental conditions and processed in parallel. Each band is representative for three experiments. Full-length gels are presented in Supplementary Fig. 6.

**Figure 5:** Effect of p50 mutant plasmid (C62S) on PL-induced cell growth inhibition and expression of Fas and DR4 in NSCLC cells as well as effect of Fas and DR4 siRNA transfection on PL induced cell growth inhibition. (**a**) Cells were transfected with p50 mutant plasmid (C62S) for 24 h, then were treated with PL (10 μM) for another 24 h. Cell viability was determined by MTT assay. Data was expressed as the mean ± S.D. of three experiments. *p < 0.05 indicates significantly different from control cells. ^#^*p* < 0.05 indicates significantly different from PL-treated cells. (**b**) Effect of p50 mutant plasmid (C62S) on the expression of DRs was determined by using Western blotting with antibodies against Fas, DR4 and β-actin (internal control). Each band is representative for three experiments. (**c**) Cells were transfected with Fas siRNA or DR4 siRNA for 24 h, and then were treated with PL (10 μM) for another 24 h. Cell viability was determined by MTT assay. Data was expressed as the mean ± S.D. of three experiments. *p < 0.05 indicates significantly different from control cells. ^#^*p* < 0.05 indicates significantly different from PL-treated cells. (**d**) Effect of Fas siRNA or DR4 siRNA transfection on DNA binding activity of NF-κB was determined by EMSA as described in the materials and methods. For the cropped images, samples were run in the same gels under same experimental conditions and processed in parallel. Full-length gels are presented in Supplementary Fig. 7.

**Figure 6:** Structure of PL and molecular binding between PL and NF-κB p50 subunit. (**a**) Structure of PL. (**b**) Pull-down assay identifies a molecular binding between PL and NF-κB p50 subunit. PL was conjugated with epoxy-activated Sepharose 4B. For the cropped images, samples were run in the same gels under same experimental conditions and processed in parallel. Full-length gels are presented in Supplementary Fig. 7. (**c,d**) Docking experiment of PL with NF-κB p50 subunit was performed as described in the materials and methods.

**Figure 7:** Anti-tumor activity of PL in lung cancer xenograft mice model. (**a–c**) Growth inhibition of subcutaneously transplanted A549 xenografts mice treated with PL (2.5 mg/kg and 5 mg/kg twice a week) for 3 weeks. Xenograft mice (n = 10) were administrated intraperitoneally with 0.01% DMSO or PL (2.5 mg/kg and 5 mg/kg). Tumor burden was measured once per week using a caliper, and calculated volume length (mm) × width (mm) × height (mm)/2. Tumor weight and volume are presented as means ± S.D. (**d**) Immunohistochemistry was used to determine expression levels of H&E, PCNA, active caspase-3, NF-κB p50 subunit in nude mice xenograft tissues by the different treatments as described in the materials and methods. We also performed DAPI&TUNEL assay to assess the apoptosis rate in the nude mice xenograft tissues. Total number of cells in a given area was determined by using DAPI nuclear staining (fluorescent microscope). A green color in the fixed cells marks TUNEL-labeled cells.

**Figure 8:** Effect of PL on the expression of apotosis regulatory proteins and on the DNA binding activity of NF-κB. (**a**) Expression of DR was determined by Western blotting with antibodies against Fas, DR4 and β-actin (internal control). (**b**) Expression of apoptosis regulatory proteins was determined by Western blotting with antibodies against cleaved capase-3, cleaved caspase-8, Bax, Bcl-2 and β-actin (internal control). (**c**) Lung tumors were lysed with A buffer and C buffer. Nuclear extracts were incubated in binding reactions of ^3^^2^p-end-labeled oligo nucleotide containing the NF-κB sequence. The present EMSA results are representative for three experiments. (**d**) Cytosol proteins were used to determine the expression of IκBα, p-IκBα and β-actin (internal control). Nuclear proteins were used to determine the expression of p50, p65 and Histone H1 (internal control) in lung tumor tissues. For the cropped images, samples were run in the same gels under same experimental conditions and processed in parallel. Each band is representative for three experiments. Full-length gels are presented in Supplementary Fig. 8 and Supplementary Fig. 9.

**Table 1:** Predicted ADME of PL.

**Test**	**PL**
Molecular weight (g/mol)	317.34
Fomular	C_17_H_19_NO_5_
Lipinski’s Rule Violations	0
Lead-like Rule Violations	0
logP	1.63
Water solubility in pure water	0.48 mg/mL
DMSO Solubility	>20 mM
Caco2 cells Permeability (×10^6^ cm/sec)	204
Human intestinal absorption (HIA, %)	100
Blood-brain barrier (BBB)	−2.20
CNS Score	−2.47
Plasma Protein Binding (% PPB)	81.00
Estrogen Receptor Binding	LogRBA < −3
hERG inhibitor probability	0.34
P-gp inhibitor probability	0.09

**Table 2:** Predicted toxicities of PL.

**Test**	**PL**
Ames Mutagenicity	0.28
Acute Tox LD_50_ (Mouse), Oral	>1,000 ml/kg
Acute Tox LD_50_ (Mouse), Intravenous	50–200 mg/kg
Irritation, Skin	0.29
Irritation, Eye	0.34
Health Effects (Probability), Gastrointestinal	0.2 < p < 0.8
Health Effects (Probability), Lung	0.2 < p < 0.8
Health Effects (Probability), Cardiovascular	p > 0.8
Health Effects (Probability), Liver	p > 0.8
Health Effects (Probability), Blood	p > 0.8
Health Effects (Probability), Kidney	0.2 < p < 0.8
Genetic toxicity	0 (negative)
Carcinogenicity	0 (negative)
Reproductive toxicity	0 (negative)

**Table 3:** Effect of PL analogues on NF-κB luciferase activity and cell growth in A549 NSCLC cells.

**No.**	**Compound name**	**IC**_**50**_ **value on NF-κB binding Activity (μM)**	**IC**_**50**_ **value on cell growth inhibition (μM)**
	Piperlongumine	1.76	14.91
1	3-phenyl-1-(piperidin-1-yl)prop-2-en-1-one	4.99	>20
2	3-(benzo-1,3-dioxol-5-yl)-1-(piperidin-1-yl)prop-2-en-1-one	5.11	>20
3	1-(piperidin-1-yl)-3-(3,4,5-trimethoxyphenyl)prop-2-en-1-one	2.68	>20
4	1-(4-methylpiperidin-1-yl)-3-phenylprop-2-en-1-one	4.39	>20
5	3-(benzo-1,3-dioxol-5-yl)-1-(4-methylpiperidin-1-yl)prop-2-en-1-one	3.39	>20
6	1-(4-methylpiperidin-1-yl)-3-(3,4,5-trimethoxyphenyl)prop-2-en-1-one	2.37	>20
7	1-(3-methylpiperidin-1-yl)-3-phenylprop-2-en-1-one	3.85	>20
8	3-(benzo-1,3-dioxol-5-yl)-1-(3-methylpiperidin-1-yl)prop-2-en-1-one	4.73	>20
9	1-(3-methylpiperidin-1-yl)-3-(3,4,5-trimethoxyphenyl)prop-2-en-1-one	3.42	>20
10	1-(2-methylpiperidin-1-yl)-3-phenylprop-2-en-1-one	5.40	18.82
11	3-(benzo-1,3-dioxol-5-yl)-1-(2-methylpiperidin-1-yl)prop-2-en-1-one	4.90	>20
12	1-(2-methylpiperidin-1-yl)-3-(3,4,5-trimethoxyphenyl)prop-2-en-1-one	2.79	>20
13	1-(2,6-dimethylpiperidin-1-yl)-3-phenylprop-2-en-1-one	3.78	>20
14	3-(benzo-1,3-dioxol-5-yl)-1-(2,6-dimethylpiperidin-1-yl)prop-2-en-1-one	5.24	>20
15	1-(2,6-dimethylpiperidin-1-yl)-3-(3,4,5-trimethoxyphenyl)prop-2-en-1-one	3.67	>20
16	1-cinnamoylpiperidin-2-one	5.56	>20
17	(E)-1-(3-(benzo-1,3-dioxol-5-yl)acryloyl)piperidin-2-one	6.06	>20
18	(E)-1-(3-(3-(3,4,5-trimethoxyphenyl)acryloyl)piperidin-2-one	3.83	>20
19	(E)-3-phenyl-1-(piperazin-1-yl)prop-2-en-1-one	3.23	19.88
20	(E)-3-(benzo[d][1,3]dioxol-5-yl)-1-(piperazin-1-yl)prop-2-en-1-one	2.67	16.20
21	(E)-1-(piperazin-1-yl)-3-(3,4,5-trimethoxyphenyl)prop-2-en-1-one	1.89	>20
22	(E)-1-(4-methylpiperazin-1-yl)-3-phenylprop-2-en-1-one	1.94	>20
23	(E)-3-(benzo[d][1,3]dioxol-5-yl)-1-(4-methylpiperazin-1-yl)prop-2-en-1-one	2.47	>20
24	(E)-1-(4-methylpiperazin-1-yl)-3-(3,4,5-trimethoxyphenyl)prop-2-en-1-one	2.17	>20
25	(E)-1-(2,6-dimethylpiperazin-1-yl)-3-phenylprop-2-en-1-one	2.78	>20
26	(E)-3-(benzo[d][1,3]dioxol-5-yl)-1-(2,6-dimethylpiperazin-1-yl)prop-2-en-1-one	2.91	>20
27	(E)-1-(2,6-dimethylpiperazin-1-yl)-3-(3,4,5-trimethoxyphenyl)prop-2-en-1-one	2.93	>20
28	(E)-1-morpholine-3-phenylprop-2-en-1-one	3.81	>20
29	(E)-3-(benzo[d][1,3]dioxol-5-yl)-1-morpholinoprop-2-en-1-one	3.79	>20
30	(E)-1-morpholino-3-(3,4,5-trimethoxyphenyl)prop-2-en-1-one	3.40	>20
31	(E)-3-phenyl-1-thiomorpholinoprop-2-en-1-one	3.45	>20
32	(E)-3-(benzo[d][1,3]dioxol-5-yl)-1-thiomorpholinoprop-2-en-1-one	4.90	>20
33	(E)-1-thiomorpholino-3-(3,4,5-trimethoxyphenyl)prop-2-en-1-one	2.20	>20
34	(E)-1-(3-methylpiperazin-1-yl)-3-phenylprop-2-en-1-one	3.80	>20
35	(E)-3-(benzo[d][1,3]dioxol-5-yl)-1-(3-methylpiperazin-1-yl)prop-2-en-1-one	3.27	>20
36	(E)-1-(3-methylpiperzain-1-yl)-3-(3,4,5-trimethoxyphenyl)prop-2-en-1-one	3.49	>20
